# Effect of Continuous Subcutaneous Injection of Insulin Analogues in Pregnant Women with Diabetes Mellitus Complicated with Ketoacidosis

This article has been retracted.

**DOI:** 10.1155/2021/8670474

**Published:** 2021-12-15

**Authors:** Yunfei Pan, Qi Wang, Feimin Zhao, Jiaying Shen, Xiaojing Zhong

**Affiliations:** ^1^General Medicine Department, Huzhou Central Hospital, Affiliated Central Hospital Huzhou University, Huzhou, China; ^2^Infectious Disease Department, Huzhou Central Hospital, Affiliated Central Hospital Huzhou University, Huzhou, China; ^3^Endocrinology Department, Huzhou Central Hospital, Affiliated Central Hospital Huzhou University, Huzhou, China

## Abstract

**Objective:**

To investigate the clinical effect of continuous subcutaneous injection of insulin analogues in pregnant women with diabetes mellitus complicated with ketoacidosis.

**Methods:**

A total of 92 pregnant patients with diabetes mellitus complicated with ketoacidosis from June 2014 to January 2021 were selected. All patients were randomly divided into an observation group and control group according to the method of random number. The control group received intravenous infusion of insulin, and the observation group received continuous subcutaneous infusion of quick-acting insulin analogues. The clinical effects of the two groups were observed.

**Results:**

The time needed to control blood glucose <13.8 mmol/L, the amount of insulin needed to control blood glucose <13.8 mmol/L, the time needed to correct DKA, and the amount of insulin needed to correct DKA in the observation group were significantly less than those in the control group (*P* < 0.05). Compared with the control group, the average occurrence times of hypoglycemia, the length of stay, the total amount of insulin in hospital, and the total amount of insulin used during pregnancy in the observation group were significantly less than those in the control group (*P* < 0.05). The values of SCr, CRP, BUN, arterial blood gas pH, and adiponectin in the two groups were significantly improved as compared with those before treatment, and the improvement in the observation group was significantly better than that in the control group (*P* < 0.05). After treatment, the fasting blood glucose, 2-hour postprandial blood glucose, carbon dioxide binding capacity, and glycosylated hemoglobin in the experimental group were significantly better than those in the routine group, and the difference was statistically significant (*P* < 0.05).

**Conclusion:**

Continuous subcutaneous injection of insulin analogues is effective in the treatment of diabetic patients with ketoacidosis, which can effectively improve blood glucose, carbon dioxide binding capacity, and glycosylated hemoglobin and accelerate the negative conversion of urinary ketone body. It is worth popularizing to reduce the occurrence of hypoglycemia and the dose of insulin and shorten the time of hospitalization.

## 1. Introduction

Ketoacidosis is a serious complication of diabetes. If it is not treated in time, it has a high mortality rate [1]. Pregnancy complicated with diabetic ketoacidosis (DKA) is an acute metabolic syndrome that can endanger the lives of pregnant women and fetuses. It usually occurs in patients with type 1 (insulin dependent) diabetes [2]. It is reported in the literature that the incidence rate is about 0.5% and 3%. DKA, which occurs during pregnancy, does great harm to the mother and fetus and can endanger their lives [3, 4]. Metabolic changes that occur during pregnancy can make pregnant diabetics more inclined to DKA [5]. At present, prenatal diabetes screening, regular prenatal examination, and positive and correct treatment have greatly improved the incidence and prognosis of ketoacidosis during pregnancy, and the maternal mortality has decreased significantly [6, 7]. However, compared with nonpregnancy, pregnancy complicated with DKA can occur when blood sugar slightly increases, and the disease progresses rapidly, which often leads to delayed diagnosis and delayed treatment; perinatal mortality is still as high as 35%–90%, and the long-term complications of surviving offspring are also high [8, 9].

Subcutaneous injection of insulin is a common scheme for the disease, but it can lead to hypoglycemia and the effect of glucose control is not ideal [10]. Quick-acting insulin analogues are a new type of insulin preparation used in clinic in recent years [11]. Insulin analogues, also known as intraprandial insulin, refer to substances that modify the structure of insulin, mimic normal insulin secretion and its normal physiological function, and are injected subcutaneously several times an hour. It is usually used in diabetes that needs insulin treatment. It has quick effect and short duration, can quickly control blood sugar in the normal range, and can reduce the level of hemoglobin at the same time. The risk of hypoglycemia is small [12], and it is also beneficial for diabetic patients to simulate the process of insulin metabolism under the physiological state of people with normal blood glucose levels [13, 14]. At present, available insulin analogues are widely used in the treatment of diabetic ketoacidosis. The commonly used insulin therapy is effective and the speed of reducing blood sugar is good, but a large amount of insulin leads to hyperinsulinemia and weight gain, and reducing the dosage of insulin can reduce the cost of treatment and shorten the duration of hospitalization. In this study, patients with diabetes mellitus complicated with ketoacidosis pregnancy were treated with continuous subcutaneous injection of insulin analogues; it accelerates the negative conversion of urinary ketone body, reduces the occurrence of hypoglycemia and the dose of insulin, and shortens the duration of hospitalization and achieved good results.

## 2. Methods

### 2.1. Study Design and Participants

A total of 92 pregnant patients with diabetes mellitus complicated with ketoacidosis from June 2014 to January 2021 were selected. All patients were randomly divided into an observation group and control group, and all the subjects received informed consent. The ethics committee of our hospital approved this research plan. All participants underwent a complete medical history examination and clinical examination.

After admission, patients in both groups were bedridden under the guidance of medical staff and received routine treatment such as anti-infection, fluid replacement, nutritional support, and maintenance of water electrolytic medium balance. The control group received intravenous infusion of insulin, which was specially filled with Nuohe Rui30 (asparagus insulin 30 injection). The product was mixed with 0.9% sodium chloride solution and injected intravenously at the rate of 0.1 U/(kg h). During the treatment, the blood glucose level of the patients was monitored in real time. When the blood glucose level dropped below 13.9 mmol/L, insulin +5% glucose solution injection was given. In the observation group, continuous subcutaneous infusion of quick-acting insulin analogues was given by subcutaneous needle embedding for 24 hours with the initial dose of 0.5 U/h, the infusion was performed during meals, and the blood glucose level of the patients was monitored. On this basis, the basic dose and infusion volume were adjusted for a total of one week.

### 2.2. Observation Index

During ketoacidosis, blood glucose at the fingertips (Lokang II blood glucose meter, produced by Roche, Switzerland), urinary ketone body, and arterial blood pH were measured every 2 hours, and the time needed to control blood glucose <13.8 mmoI/L (h), the negative time of urinary ketone body, the dose of insulin needed to correct diabetic ketoacidosis, the average occurrence of hypoglycemia, and the length of hospital stay were observed. The levels of creatinine (SCr), serum C-reactive protein (CRP), urea nitrogen (BUN), arterial blood gas pH, and adiponectin were observed and compared between the two groups before treatment and 1 week after treatment. The differences of fasting blood glucose, 2-hour postprandial blood glucose, carbon dioxide binding capacity, and glycosylated hemoglobin between patients before and after treatment were observed.

### 2.3. Inclusion and Exclusion Criteria

Inclusion criteria: (1) clinical symptoms and signs meet the diagnostic criteria of diabetic ketoacidosis; (2) there is no contraindication of quick-acting insulin analogues; (3) age is not less than 18 years; and (4) patients understand the details of the study and participate actively. Exclusion criteria: (1) patients with impaired function of important organs and poor stability of vital signs; (2) those who were treated with other treatments at the present stage; and (3) those complicated with other types of endocrine or immune system diseases.

### 2.4. Statistical Analysis

The data were analyzed by SPSS25.0 statistical software, and the clinical data (measurement data) were expressed as mean ± standard deviation ($\bar{x}$ ± *S*). One-way ANOVA was used for comparison between groups. A paired *t* test was used for intragroup comparison, independent-sample *t* test was used for intergroup comparison, counting data were expressed as rate (%), and *χ*^2^ test was performed, and the difference was statistically significant (*P* < 0.05).

## 3. Result

A total of 349 pregnant patients with diabetes mellitus complicated with ketoacidosis were treated in our hospital from June 2014 to January 2021.167 patients did not meet the inclusion and exclusion criteria, and 90 patients refused to participate. A total of 92 patients were randomly divided into an observation group (*n* = 46) and control group (*n* = 46), as shown in Figure 1.

The age of the observation group was 24–38 years, the average age was 29.4 ± 8.5 years, the BMI: 25.74 ± 1.63, the age of the patients in the control group was 22–36 years, the average age was 28.9 ± 9.1 years, and BMI: 25.69 ± 1.88. There was no significant difference in the condition, course of disease, and other general data of the selected patients (*P* > 0.05). See Table 1 for details.

### 3.1. Comparison of the Time Needed to Control Blood Glucose <13.8 mmol/L, the Amount of Insulin Needed to Control Blood Glucose <13.8 mmol/L, the Time Needed to Correct DKA, and the Amount of Insulin Needed to Correct DKA

The time needed to control blood glucose <13.8 mmol/L, the amount of insulin needed to control blood glucose <13.8 mmol/L, the time needed to correct DKA, and the amount of insulin needed to correct DKA in the observation group were significantly less than those in the control group, *P* < 0.05, see Table 2.

### 3.2. The Average Occurrence of Hypoglycemia, the Length of Stay, the Total Dosage of Insulin during Hospitalization, and the Total Amount of Insulin Used during Pregnancy Compared between the Two Groups

Compared with the control group, the average occurrence times of hypoglycemia, the length of stay, the total amount of insulin in hospital, and the total amount of insulin used during pregnancy in the observation group were significantly less than those in the control group (*P* < 0.05), as shown in Table 3.

### 3.3. Comparison of Creatinine SCr, CRP, BUN, Arterial Blood Gas pH, and Adiponectin between the Two Groups before and after Treatment

There was no significant difference in SCr, CRP, BUN, arterial blood gas pH, and adiponectin between the two groups, but after treatment, SCr, CRP, BUN, arterial blood gas pH, and adiponectin in the two groups were significantly improved compared with those before treatment (*P* < 0.05), and the improvement in the observation group was significantly better than that in the control group (*P* < 0.05), see Table 4.

### 3.4. Comparison of Fasting Blood Glucose, 2-Hour Postprandial Blood Glucose, Carbon Dioxide Binding Capacity, and Glycosylated Hemoglobin before and after Treatment

Before treatment, fasting blood glucose, 2-hour postprandial blood glucose, carbon dioxide binding capacity, and glycosylated hemoglobin were similar between the two groups, but there was no significant difference between the two groups (*P* > 0.05). After treatment, the improvement of fasting blood glucose, 2-hour postprandial blood glucose, carbon dioxide binding capacity, and glycosylated hemoglobin in the experimental group was more significant than that in the routine group, and the difference was statistically significant (*P* < 0.05), see Table 5.

## 4. Discussion

DKA is one of the internal medical emergencies, which refers to the syndrome caused by abnormal metabolism of sugar, protein, and fat caused by the deficiency of hormones and the increase of insulin reverse hormone in the human body [12, 15]. At the same time, common and multiple complications in patients with type 1 diabetes can also occur in the stress state of type 2 diabetes. Diabetes mellitus complicated with ketoacidosis will seriously threaten the life safety of pregnant women and newborns [16, 17]. Patients with mild ketoacidosis usually have symptoms such as elevated blood sugar, polyuria, abnormal breathing, headache, oliguria, and moderate and severe gestational diabetes with ketoacidosis. There will be pupil fixation, breathing with rotten apple odor, and nausea and vomiting symptoms [18–20]. If the patient has ketoacidosis, the risk of intrauterine death, neonatal asphyxia, and hyperbilirubinemia will occur, which will seriously affect the normal growth and development of the fetus [21]. In addition, gestational diabetes mellitus complicated with ketoacidosis can cause fetal congenital malformation, intrauterine distress, etc. and may also lead to maternal hypertension, polyhydramnios, and infection [22–24]. The occurrence of DKA is related to infection, operation, trauma, improper diet, improper use of insulin, and cardiocerebrovascular disease [25]. Gestational diabetic ketoacidosis will have a great impact on the quality of life of patients and the safety of maternal and infant life, and with the increase of gestational weeks, the level of insulin in patients will also be greatly increased; therefore, to explore the effective treatment of gestational diabetic ketoacidosis has a very important clinical value [26, 27]. In the treatment of gestational diabetic ketoacidosis, clinical drug treatment is mainly used, such as sodium chloride injection expansion, potassium supplement, and insulin drip [28, 29].

Insulin analogues can enable patients with diabetes to achieve better blood glucose goals, with a lower incidence of hypoglycemia and a better quality of life than short- and long-acting human insulin [30, 31]. Previous studies have pointed out that when pregnancy patients complicated with DKA are treated with insulin-like drugs, the risk of hypoglycemia events is reduced, the allergic reaction is less, and the reaction at the injection site is reduced. It has the potential to promote mitosis and the safety of medication during pregnancy. For patients prone to severe hypoglycemia, the use of complete insulin analogues can lead to rapid cost savings, so insulin analogues should be the standard treatment for all patients with type 1 diabetes [32]. The new long-acting insulin analogues glargine U300 insulin and hypoglycemic insulin have been shown to be more stable, which can reduce the risk of nocturnal hypoglycemia and increase the flexibility of administration time [33, 34]. Insulin analogues enable patients to live an active life without sacrificing strict blood sugar control [35]. This study showed that the time needed to control blood glucose <13.8 mmol/L, the amount of insulin needed to control blood glucose <13.8 mmol/L, the time needed to correct DKA, and the amount of insulin needed to correct DKA in the observation group were significantly less than those in the control group (*P* < 0.05). Compared with the control group, the average occurrence times of hypoglycemia, the length of stay, the total amount of insulin in hospital, and the total amount of insulin used during pregnancy in the observation group were significantly less than those in the control group (*P* < 0.05). The values of SCr, CRP, BUN, arterial blood gas pH, and adiponectin in the two groups were significantly improved as compared with those before treatment, and the improvement in the observation group was significantly better than that in the control group (*P* < 0.05). Fasting blood glucose, 2-hour postprandial blood glucose, carbon dioxide binding capacity, and glycosylated hemoglobin were significantly improved (*P* < 0.05). It is suggested that continuous subcutaneous injection of insulin is effective in the treatment of diabetic patients with ketoacidosis, which can effectively improve blood glucose, carbon dioxide binding capacity, and glycosylated hemoglobin, accelerate the negative conversion of urinary ketone body, reduce the occurrence of hypoglycemia and insulin dose, and shorten the length of stay.

In summary, the treatment of continuous subcutaneous injection of insulin-like drugs in patients with gestational diabetes mellitus with ketoacidosis can improve patient indicators, reduce maternal and infant risk, shorten hospital stay, and reduce the incidence of adverse events, which is worth popularizing.

## Figures and Tables

**Figure 1:** Flow chart of inclusion and exclusion of patients.

**Table 1:** Baseline characteristics of participants.

	Observation group (*N* = 46)	Control group (*N* = 46)
Age (years)	29.4	28.9
Duration of diabetes (years)	3.39	3.48
HbA1c above 75 mmol/mol (9.0%) (%)	28 (61.7%)	32 (70.0%)
Average number of hypoglycemic (<3.88 mmol/L) episodes lasting 15 or more minutes per 24 hr period	0.47 (0.86)	0.45 (0.8)
BMI	25.74 ± 1.63	25.69 ± 1.88
Total cholesterol (mmol/L)	4.27 (0.83)	4.21 (0.86)
LDL cholesterol (mmol/L)	2.37 (0.67)	2.35 (0.6)
HDL cholesterol (mmol/L)	1.32 (0.21)	1.32 (0.24)
Triglycerides (mmol/L)	0.88 (0.43)	1.10 (2.22)
Systolic blood pressure (mmHg)	101 (9)	102 (9)
Diastolic blood pressure (mmHg)	66 (7)	67 (9)

**Table 2:** Comparison of the time required to control blood glucose <13.8 mmol/L, the amount of insulin required for blood glucose <13.8 mmol/L, the time required to correct DKA, and the amount of insulin required to correct DKA ($\bar{x}$ ± *S*).

	Observation group	Control group	*P*
The time required to control blood glucose <13.8 mmol/L	6.5 ± 1.3	7.2 ± 1.5	0.019
The amount of insulin required for blood glucose <13.8 mmol/L	55.9 ± 4.5	58.32 ± 4.9	0.016
The time required to correct DKA	14.6 ± 2.0	19.4 ± 2.3	<0.001
The amount of insulin required to correct DKA	88.4 ± 5.7	83.3 ± 6.4	<0.001

**Table 3:** Comparison of the average occurrence times of hypoglycemia, the length of stay, the total dosage of insulin during hospitalization, and the total amount of insulin used during pregnancy between the two groups.

	Observation group	Control group	*P*
The average occurrence of hypoglycemia	0.90 ± 0.27	2.85 ± 0.63	<0.001
The length of stay (d)	9.13 ± 2.95	14.01 ± 3.77	<0.001
The total dosage of insulin during hospitalization	126.4 ± 7.9	171.3 ± 8.4	<0.001
The total amount of insulin used during pregnancy	298.39 ± 64.61	361.76 ± 75.44	<0.001

**Table 4:** Comparison of creatinine SCr, CRP, BUN, arterial blood gas pH, and adiponectin between the two groups before and after treatment.

Groups		SCr (umol/L)	CRP (mg/L)	BUN (mmol/L)	Arterial blood gas pH	Adiponectin (ug/L)
Observation group	Before treatment	187.02 ± 14.79	13.85 ± 4.17	15.23 ± 3.84	6.79 ± 1.20	6.38 ± 1.41
Control group		186.93 ± 15.42	13.82 ± 5.94	15.31 ± 3.90	6.98 ± 2.11	6.40 ± 1.39
Observation group	After treatment	132.05 ± 12.94^ab^	3.39 ± 3.10^ab^	8.64 ± 1.67^ab^	7.55 ± 0.48^ab^	15.87 ± 3.03^ab^
Control group		151.16 ± 12.51^a^	7.47 ± 2.22^a^	10.72 ± 1.21^a^	7.04 ± 0.43^a^	10.28 ± 2.19^a^

Note: compared with before treatment, ^a^*P* < 0.05; compared with the routine group after treatment, ^b^*P* < 0.05.

**Table 5:** Comparison of fasting blood glucose, 2-hour postprandial blood glucose, carbon dioxide binding capacity, and glycosylated hemoglobin before and after treatment.

Groups		Fasting blood glucose	2-hour postprandial blood glucose	Carbon dioxide binding capacity	Glycosylated hemoglobin (%)
Observation group	Before treatment	18.73 ± 4.27	23.59 ± 4.29	16.79 ± 3.72	12.53 ± 1.61
Control group		18.96 ± 5.61	23.57 ± 4.19	16.86 ± 3.62	12.82 ± 1.29
Observation group	After treatment	8.81 ± 1.17^ab^	9.32 ± 1.95^ab^	25.85 ± 3.62^ab^	7.30 ± 1.45^ab^
Control group		10.34 ± 3.92^a^	14.13 ± 3.49^a^	20.82 ± 2.21^a^	9.74 ± 1.87^a^

Note: compared with before treatment, ^a^*P* < 0.05; compared with the routine group after treatment, ^b^*P* < 0.05.

## Data Availability

The simulation experiment data used to support the findings of this study are available from the corresponding author upon request.
